The article "Diagnosis and Etiological Analysis of Gastroesophageal Reflux Disease by Gastric Filling Ultrasound and GerdQ Scale" was retracted in 2023. Reasons: signs of a paper mill; suspected computer-generated content; unreliable results or conclusions; lack of ethics approval or compliance.

# Diagnosis and Etiological Analysis of Gastroesophageal Reflux Disease by Gastric Filling Ultrasound and GerdQ Scale

**DOI:** 10.1155/2021/5629067

**Published:** 2021-11-15

**Authors:** Bo Wang, Qian Sun, Yonghong Du, Kexiao Mu, Jingxia Jiao

**Affiliations:** ^1^Department of Physical Diagnostics, West Hospital District of Qingdao Multicipal Hospital, Qingdao 266002, China; ^2^Department of Ultrasound, the Second Affiliated Hospital of Shandong University of Traditional Chinese Medicine, Jinan 250000, China

## Abstract

**Objective:**

To investigate the diagnosis and etiological analysis of GERD by gastric filling ultrasound and GerdQ scale.

**Methods:**

The clinical data of 100 suspected GERD patients were selected for retrospective analysis. The selection time was from June 2016 to June 2019. According to the gold standard (endoscopy) results, they were divided into the gastroesophageal reflux group (positive, *n* = 62) and the nongastroesophageal reflux group (negative, *n* = 38); both gastric filling ultrasound and GerdQ scale examination were performed to compare the positive predictive value and negative predictive value, evaluate the abdominal esophageal length, His angle, and GerdQ scale score, and analyze the AUC value, sensitivity, specificity, and Youden index of His angle, length of abdominal esophagus, combined ultrasound parameters, and GerdQ scale in the diagnosis of GERD.

**Results:**

100 patients with suspected GERD were diagnosed as GERD by endoscopy; in a total of 62 cases, the percentage was 62.00%. Among them, 28 cases were caused by the abnormal structure and function of the antireflux barrier, accounting for 45.16%, 18 cases were caused by the reduction of acid clearance of the esophagus, accounting for 29.03%, and 16 cases were caused by the weakening of the esophageal mucosal barrier, accounting for 25.81%. After ultrasound detection, the positive predictive value was 88.71% and the negative predictive value was 81.58%; after the GerdQ scale was tested, the positive predictive value was 71.43% and the negative predictive value was 54.05%. The length of the abdominal esophagus in the gastroesophageal reflux group was lower than that of the nongastroesophageal reflux group, while the scores of His angle and GerdQ scale were higher than those in the gastroesophageal reflux group (*P* < 0.05). ROC curve analysis showed that the AUC values of His angle, length of abdominal esophagus, combined ultrasound parameters, and GerdQ scale to diagnose GERD were 0.957, 0.861, 0.996, and 0.931 (*P* < 0.05), their sensitivity was 93.5%, 98.40%, 98.40%, and 90.30%, and the specificity was 92.10%, 63.20%, 100.00%, and 92.10%, respectively.

**Conclusion:**

Both gastric filling ultrasound and GerdQ scale have a certain application value in the diagnosis of GERD, but the former has a higher accuracy rate, and it is more common for gastroesophageal reflux caused by abnormal structure and function of antireflux barrier in etiological analysis.

## 1. Introduction

Gastroesophageal reflux disease (GERD) is a functional disease caused by the reflux of duodenal contents into the esophagus with lesions of esophageal mucosa and extraesophageal tissues [1]. The clinical manifestations of the disease are complex and varied, with acid reflux, antifeeding, and burning pain under xiphoid or substernum as the typical clinical symptoms. In patients with obvious clinical manifestations, the diagnosis can be made by typical symptoms, but there are also some patients with atypical clinical symptoms; in this case, the use of auxiliary examination is particularly important. The most reliable method for the diagnosis of gastroesophageal reflux and gastroesophageal reflux disease is 24-hour pH detection, which can not only detect reflux but also understand the relationship between the degree of reflux and symptoms, body position, and feeding. However, the application of the pH detection method is limited because it has not been widely used in China [2]. At present, the diagnosis of gastroesophageal reflux disease in China uses a combination of clinical, endoscopic, and physiological parameters. Based on the inner diameter manifestations of esophagitis, long Barrett's esophagus, or digestive stenosis, the diagnosis of pathological reflux esophageal connective tissue can be made [3]. Clinically, endoscopy is regarded as the golden standard for the diagnosis of this disease. However, as this method is invasive and intolerable for some patients and is not suitable for promotion in primary hospitals [4], it is very important to find a noninvasive examination method with high accuracy. The GerdQ scale has been suggested by clinical scholars for examination. The GerdQ scale was found by Dent et al. in 2007 and optimized by three scales called Reflux Disease Questionnaire (RDQ), Gastroesophageal Reflux Disease Impact Scale (GIS), and Gastrointestinal Symptom Grade Scale (GSRS), widely used in clinical practice [5, 6], At the same time, some scholars suggest the use of ultrasound examination. However, there are few comparative studies on the above two methods, and it is not clear which method has high accuracy and specificity. Therefore, the clinical data of 100 suspected GERD patients were selected for retrospective analysis in order to discuss the diagnosis of GERD by gastric filling ultrasound and GerdQ scale and analyze its etiology. They are now reported in the following.

## 2. Data and Methods

### 2.1. Clinical Data

Clinical data of 100 suspected GERD patients diagnosed and treated from June 2016 to June 2019 were retrospectively analyzed. Diagnostic criteria: the diagnosis was confirmed by esophageal reflux monitoring and upper gastrointestinal endoscopy in accordance with the diagnostic criteria of “multidisciplinary diagnosis and treatment consensus of gastroesophageal reflux disease in China” [7]. Inclusion criteria:(1) age ≥18 years; (2) at least one of the clinical manifestations such as reflux, acid reflux, or heartburn in the past 4 weeks. Exclusion criteria:(1) recent dysphagia, weight loss, and other symptoms; (2) after physical examination, there are abnormalities such as rebound pain and mass in the abdomen; and (3) accompanied by serious heart, liver, kidney, and other diseases. There was no significant difference in general data between the two groups (*P* > 0.05), as given in Table 1.

### 2.2. Methods

The data of 100 patients with suspected GERD undergoing ultrasound examination and GerdQ scale assessment were retrospectively analyzed.

#### 2.2.1. Ultrasonic Detection Method

Color Doppler ultrasound diagnostic instrument is produced by Siemens GE 4D convex array probe, probe frequency of 3.5–5.5 mhz. Pretest routine fasting should be 8–12 h and 5 min before testing guide patients with oral gastric ultrasound help agent 500 ml, guide the patient to sitting, dynamic scan end of the esophagus and cardia, gastric, gastric body, gastric antrum, pylorus, duodenum, and observe whether the stomach wall form changes, changes of peristaltic frequency, contents emptying condition, the existence of a reverse flow, echo property, and vascular distribution of lesion were recorded. Then, assist the patient to take the supine position, select the oblique section of the left costal margin under the xiphoid process, instruct the patient to maintain the breath-holding state after forcibly inhaling, put the probe toward the left lobe of the liver septum, and gently press the abdominal wall. The angle between the parallel line of the long axis of the feeding tube and the tangent line of the fundus of the stomach was His angle. The distance between the esophageal hiatus and the place was taken as the length of the abdominal esophagus, and the mean value was taken as the final result.

#### 2.2.2. Gastroesophageal Reflux Disease Questionnaire (GerdQ) Scale [8]

The scale was used to assess the patients' symptoms in the last week, The assessment included 6 items, including frequency of reflux attacks, frequency of gastric burning attacks, frequency of nausea, frequency of upper abdominal pain, frequency of self-medication for sleep disorders, and frequency of using OTC drugs. The frequency of nausea and the frequency of upper abdominal pain are assessed inversely, that is, 0 d is 3 points, 1 d is 2 points, 2-3 d is 1 point, and 4–7 d is 0 points; the others are positive scores, that is, 0 d is 0 point, 1 d is 1 point, 2-3 d is 2 points, and 4–7 d is 3 points. Finally, the total score of 6 items ≥8 points is judged as positive, that means suffering from GERD.

### 2.3. Observation Index

  The positive predictive value and negative predictive value of 100 subjects were measured by ultrasound and GerdQ scale, using the four-cell table method
  The length of abdominal esophagus, His angle, and GerdQ scale scores of 2 groups were evaluated
  His angle, abdominal esophageal length, combined ultrasound parameters, AUC value, sensitivity, specificity, and Youden index of GERD were evaluated. Combined ultrasound parameters = abdominal esophagus length + (*β* His angle/*β* abdominal esophagus length) × His angle, where *β* was used as the dependent variable, and abdominal esophagus length and His angle were used as independent variables to carry out the regression coefficient of binary logistic regression.

### 2.4. Statistical Method

SPSS22.0 software was used to analyze the data. Measurement data were represented by ($\bar{x}\pm s$), and the independent sample *T*-test was performed. Counting data were represented by (*n*; %), the *χ*^2^ test was performed. The predictive value was analyzed by the ROC curve. *P* < 0.05 was considered as a statistically significant difference.

## 3. Result

### 3.1. Etiological Analysis

Among the 100 suspected GERD patients, 62 cases (62.00%) were confirmed to be GERD by endoscopic examination. Among them, 28 cases (45.16%) were caused by the abnormal structure and function of antireflux barrier, 18 cases (29.03%) were caused by the reduced function of esophageal scavenging acid, and 16 cases (25.81%) were caused by the reduced function of esophageal mucosal barrier.

### 3.2. Comparison of Positive and Negative Predictive Values

The positive predictive value and negative predictive value of 100 suspected GERD patients were 88.71% and 81.58% after ultrasonic examination. The positive predictive value was 71.43% and the negative predictive value was 54.05%.  Table 2 provides the details.

### 3.3. Comparison of Abdominal Esophageal Length, His Angle, and GerdQ Scale Scores

The abdominal esophageal length of the GERD group was lower than that of the non-GERD ultrasound group, while His angle and GerdQ scale scores were higher than those of the GERD group (*P* < 0.05).  Table 3 provides the details.

### 3.4. Diagnostic Performance Analysis

ROC curve analysis showed that the AUC values of His angle, abdominal esophageal length, combined ultrasound parameters, and GerdQ scale for GERD diagnosis were 0.957, 0.861, 0.996, and 0.931 (*P* < 0.05). According to AUC and standard error, the difference of AUC was tested by *Z*, and the results showed that His angle vs. abdominal esophageal length *Z* = 2.26, *P*=0.024; His angle vs. ultrasonic combined parameters *Z* = −1.985, *P*=1.953; His angle vs. GerdQ scale score *Z* = 0.828, *P*=0.408; abdominal esophageal length vs. ultrasound combined parameters *Z* = −3.522, *P*=2.00; abdominal esophageal length vs. GerdQ scale score *Z* = −1.539, *P*=1.876; and ultrasound combined parameters vs. GerdQ scale score *Z* = 2.55, *P*=0.011. According to the optimal critical value, when His angle was higher than 58.135°, the sensitivity and specificity were 93.5% and 92.1%, respectively. When the length of abdominal esophagus was higher than 3.295 cm, the sensitivity and specificity were 98.4% and 63.2%, respectively. When the ultrasonic combination parameter is lower than −4.40702, the sensitivity is 98.4% and the specificity is 100%. When GerdQ score was higher than 7.31, the sensitivity and specificity were 90.3% and 92.1%, respectively.  Table 4 provides the details. ROC curves are shown in Figures 1 and 2.

## 4. Discussion

According to the epidemiological investigation [9], the prevalence of GERD is about 5.77%. The prevalence of GERD in European countries is as high as 10%–20%, while the prevalence of GERD in Asia is less than or slightly lower. In recent years, with the economic and social development, people's living habits and diet structure have been improved to some extents, the aging degree has increased, and the unhealthy lifestyle has led to the increase in the incidence of GERD. The incidence of disease will be increasing with people's living habits and diet structure [10]. Clinically, it is believed that the occurrence of this disease is related to the abnormal structure and function of the antireflux barrier, the reduced function of esophageal acid clearance, and the weakened role of esophageal mucosal barrier [11–13]; at the same time, esophageal mucosa inflammation and motor disorders are also associated with the severity of GERD [14]. Previous studies have shown that the proportion of GERD caused by the first etiology is the highest, and the abnormal structure and function of the antireflux barrier are mostly related to dietary habits and living habits, such as obesity, which lead to the damage of the lower esophageal sphincter structure by promoting the increase of abdominal pressure [15]. Studies have also pointed out that long-term use of calcium channel blockers, aminophylline, diazepam, and other drugs will also cause esophageal motor dysfunction and lower esophageal sphincter pressure drop [16]. Studies have also pointed out that long-term use of calcium channel blockers, aminophylline, diazepam, and other drugs will also cause esophageal motor dysfunction and lower esophageal sphincter pressure drop. The above research results indicate that maintaining good living habits and eating habits is particularly important to reduce the incidence of GERD. In the past, X-ray barium meal examination was mostly used for clinical diagnosis of this disease, which provided important information for clinical diagnosis by comprehensively observing the shape of the stomach, length of the abdominal cavity and esophagus, His angle, and frequency of gastroesophageal reflux. However, due to the limitation of instantaneous performance, it was difficult to distinguish physiological reflux from pathological reflux. Some studies have pointed out that the reflux rate detected by X-ray barium meal in normal population is about 20% or even higher, while the detection rate in the diagnosis of pathological acid reflux is only 26%, indicating its low sensitivity and specificity [17]. With the further development of imaging technology, clinical ultrasound examination of GERD can not only dynamically and intuitively observe esophageal peristalsis, length of abdominal esophagus, His angle, and other information but also measure gastric empty. With advantages of good repeatability, simple operation, and convenience, it has been widely used and promoted in clinical practice [18].

The results of this study showed that the positive predictive value and negative predictive value of GERD in gastric filling ultrasound diagnosis were 88.71% and 81.58%, respectively. The results are close to the gold standard. In addition, when measuring the length of the abdominal esophagus and His angle, it was found that the length of the abdominal esophagus in the GERD group was shorter than that in the non-GERD group, while His angle was higher than that in the non-GERD group, which may be related to the anatomical abnormalities of the lower gastroesophageal segment. Under normal circumstances, the anatomical structure of the lower segment of the stomach and esophagus can play an antireflux role. For example, His angle connecting the esophagus and stomach is a one-way valve to prevent reflux, while the abdominal esophagus is affected by abdominal pressure and plays an antireflux role by promoting the wall of the tube to converge [19–21]. However, when His angle increases, it means that the diaphragmatic angular clamp is weakened and cannot prevent the occurrence of reflux symptoms. Studies [22] pointed out that under the stomach esophagus period of abnormal anatomical structure is a common cause of gastroesophageal reflux, and in the GERD group, it was found that the ventral segment esophageal length shorter than the general population prompt the stomach esophagus in patients with the gastroesophageal reflux period of abnormal change in anatomy, and ultrasound examination can directly observe the stomach esophagus connection department of anatomy. It can provide quantitative or semiquantitative index for the degree of reflux. Some scholars also suggest the use of the GerdQ scale, which is a newly developed new diagnostic method, and provide information for clinical diagnosis by understanding the frequency and severity of symptoms [23, 24]. However, in this study, it was found that the specificity of GERD was relatively low, so the GerdQ scale can only be used as a preliminary screening diagnostic tool. In addition, in ROC curve analysis, it was found that the AUC value of the GerdQ scale was lower than that of His angle and abdominal esophageal length, indicating that its predictive value was lower than that of ultrasound. In addition, this study proposed “ultrasound combined parameter,” that is, His angle combined with abdominal esophageal length to diagnose GERD. Its AUC value and specificity are significantly higher than His angle and abdominal esophageal length alone, indicating that combined diagnosis has a higher predictive value and can provide more accurate reference information for GERD diagnosis, thus reducing the rate of misdiagnosis and missed diagnosis.

In conclusion, both gastric filling ultrasound and the GerdQ scale have a certain application value in the diagnosis of GERD, but the diagnostic value of gastric filling ultrasound is higher, especially the combination of His angle and abdominal esophageal length can further improve the diagnosis and confirmation rate.

## Figures and Tables

**Figure 1:** ROC curve analysis of His angle and GerdQ scale scores.

**Figure 2:** ROC curve analysis of abdominal esophagus length and ultrasonic combined parameters.

**Table 1:** Comparison of general information.

Group	Gender (%)		Mean age	BMI index (kg/m^2^)
	Male	Female		
GERD (*n* = 62)	32 (51.61)	30 (48.39)	45.23 ± 3.52	22.32 ± 2.02
Non-GERD (*n* = 38)	19 (50.00)	19 (50.00)	45.28 ± 3.50	22.36 ± 1.95
*χ* ^*2*^ */t*	0.025		0.069	0.097
*P*	0.876		0.945	0.923

**Table 2:** The positive and negative predictive values of the two methods were compared.

Golden standard	Ultrasound		GerdQ		Sum
	Positive	Negative	Positive	Negative	
GERD	55	7	45	17	62
Non-GERD	7	31	18	20	38
Sum	62	38	63	37	100

*Note.* The gold standard is endoscopic examination; the GERD group was positive and the non-GERD group was negative.

**Table 3:** Comparison of abdominal esophageal length, His angle, and GerdQ scale scores between the two groups.

Group	*n*	Ultrasound		GerdQ
		Length of abdominal esophagus (cm)	His angel (°)	
GERD	62	2.36 ± 0.75	68.23 ± 6.52	8.35 ± 2.85
Non-GERD	38	3.49 ± 0.60	52.45 ± 5.09	5.75 ± 1.02
T		7.867	12.723	5.407
*P*		<0.001	<0.001	<0.001

**Table 4:** ROC curve analysis of the four detection methods.

Test result variable	AUC	Standard error	*P*	95% confidence interval		Cutoff	Youden' index	Sensitivity	Specificity
				Lower limiting value	Higher limiting value				
His angel	0.957	0.019	<0.001	0.920	0.993	58.135	0.856	93.50	92.10
Length of abdominal esophagus	0.861	0.038	<0.001	0.787	0.934	3.295	0.616	98.40	63.20
Ultrasonic combination parameter	0.996	0.005	<0.001	0.987	1.000	−4.4070	0.984	98.40	100.00
GerdQ score	0.931	0.025	<0.001	0.882	0.980	7.31	0.824	90.30	92.10

*Note.* The parameters of ultrasonic combination are His angle and abdominal esophagus length, and its formula is calculated as ultrasonic combination parameter = abdominal esophagus length + 0.360/2.791 ^*∗*^ His angle.

## Data Availability

The dataset used to support the findings of this study are available from the corresponding author upon request.
